This article has been retracted.

# Post-COVID reactivation of latent *Bartonella henselae* infection: a case report and literature review

**DOI:** 10.1186/s12879-024-09336-7

**Published:** 2024-04-22

**Authors:** Yanzhao Dong, Ahmad Alhaskawi, Xiaodi Zou, Haiying Zhou, Sohaib Hasan Abdullah Ezzi, Vishnu Goutham Kota, Mohamed Hasan Abdulla Hasan Abdulla, Alenikova Olga, Sahar Ahmed Abdalbary, Hui Lu

**Affiliations:** 1 Department of Orthopedics, The First Affiliated Hospital, Zhejiang University, #79 Qingchun Road, Hangzhou, Zhejiang Province 310003 People’s Republic of China; 2 The Second Affiliated Hospital of Zhejiang Chinese Medical University, Hangzhou, Zhejiang Province 310003 People’s Republic of China; 3 School of Biomedical Science, Faculty of Medicine, The Chinese University of Hong Kong, Rm 706, 7/F, Lo Kwee-Seong Integrated Biomedical Science Bldg, Shatin, New Territories Hong Kong, China; 4 Department of Orthopedics, Third Xiangya Hospital, Central South University, #138 Tongzi po Road, Changsha, Hunan Province 410013 People’s Republic of China; 5 Zhejiang University School of Medicine, #866 Yuhangtang Road, Hangzhou, Zhejiang Province 3100058 People’s Republic of China; 6 Department of Neurology, Republican Research and Clinical Center of Neurology and Neurosurgery, Skoriny, Minsk, Belarus; 7 Department of Orthopedic Physical Therapy, Faculty of Physical Therapy, Nahda University in Beni Suef, Beni Suef, Egypt

**Keywords:** Cat scratch disease (CSD), *Bartonella henselae*, COVID-19, High-throughput sequencing

## Abstract

Cat scratch disease (CSD) is caused by *Bartonella henselae* (*B. henselae*) and presents as lymphadenopathy following close contact with cats. However, in context of the global COVID-19 pandemic, clinical manifestations of CSD may vary, posing new challenges for healthcare professionals. Here we describe a case of a 54-year-old male with painful left upper arm mass, which gradually resolved until he was infected with COVID-19. The mass then rapidly progressed before admission. Meanwhile, pulmonary symptoms including pleural effusion emerged simultaneously. The cause was undetermined with routine blood culture and pathological test until the next generation sequencing (NGS) confirmed the presence of *B. henselae*. We believe this case is the first to report localized aggravation of CSD after COVID-19 infection and hopefully, offers treatment experience for clinicians worldwide.

## Introduction

Cat-scratch disease (CSD), an uncommon infection often observed in households with domestic cats, is first described in 1950 by Debré R. et al. [1]. The causative pathogen of CSD is *Bartonella henselae* (*B. henselae*), a Gram-negative rod that can be detected by immunohistochemistry and several silver staining methods including Warthin-Starry stain, Steiner stain and Dieterle stain [2]. At the early stage of infection, CSD normally presents as non-specific lymphadenopathy affecting both adults and children [3]. As an infectious disease, CSD has been reported worldwide and higher incidents are reported in the autumn and winter, perceivably associated the seasonal breeding of domestic cats [4].

CSD is commonly seen among young adults and children, and the major clinical manifestations of CSD include a papule at the site of microbe entrance and axillary node lymphadenopathy, which could progress to fever, aches, nausea, abdominal pain and malaise [5]. Diagnosis of CSD is usually dependent on both history of cat contact and primary lesions followed by regional lymphadenopathy, which can be further confirmed via serological evidence, blood or suppuration culture, and the next generation sequencing (NGS). However, *B. henselae* is a slow-growing bacterium, and bacterial culture could take up to 21 days, with a high false-negative rate. While serological tests could aid in the diagnosis, they often fail to differentiate between *B. henselae* and other *Bartonella* species. Furthermore, positive serological results may persist for years after treatment. In contrast, NGS is a highly accurate method for identifying various pathogens including *B. henselae*. Additionally, NGS can provide quantitative data regarding the detected pathogen, serving as an indicator of the infection’s severity. This quantitative information can be invaluable in monitoring the status of the infection. Approximately 90% of untreated lymphadenitis and lymph node enlargement following CSD gradually regress to normal size in immunocompetent patients over a period of several months, while the remaining 10% patients could progress to cutaneous erythema and result in spontaneous suppuration [6]. In these cases, the combined use of azithromycin and rifampin orally or intravenously is recommended, although the dosage and course may vary [7, 8].

While CSD is the most common manifestation of bartonellosis and over 90% cases of CSD are benign and self-limiting, the spectrum of bartonellosis is expanding as several studies and cases have elucidated association between *Bartonella* infection and cardiovascular, neurological, psychiatric, ocular and rheumatic disorders [9–13]. For immunocompromised patients, *B. henselae* infection elicits vasoproliferative responses instead of localized lymphadenopathy, and manifests as a cutaneous angiogenic lesion with inflammatory cell infiltrates [1]. What is causing this phenomenon, however, is still under debate. Moreover, disseminated bartonellosis has been observed in several cases of patients with human immunodeficiency virus (HIV) infection, and one of the cases reported rapid exacerbation to respiratory failure and ultimately, death of the patient [14–16]. As our understanding grows, it is being increasing acknowledged that bartonellosis is a major public health issue, and efforts made to better comprehend its reservoir and vector can be assimilated into solving this problem [17].

Since its discovery, CSD has been studied comprehensively by research groups across the world. Nevertheless, little is known about CSD progression in the context of Coronavirus disease 2019 (COVID) infection, with only one case report available on coinfection of COVID and *B. henselae* in 2021 [18]. We believe that this is the first case to report reactivation of *B. henselae* post COVID infection.

## Case presentation

On January 31, 2023, a previously healthy male was admitted with a one-month history of red and swollen mass on the ulnar side of left upper arm. At the onset of the swollen mass, he visited the local clinic and ultrasound (US) examination was ordered, indicating inflammation with abscess formation. Therefore, he was prescribed with oral administration of cefuroxime (250 mg, BID) for 7 days and pain relief treatment (irecoxib, 100 mg, BID). The mass gradually resolved until shortly progression complicated with symptoms of fever (Tmax = 39.5 °C), cough, fatigue, myalgia, shortness of breath and anorexia, which was confirmed to be COVID infection by local hospital. During this period, he observed rapid progression of the original mass with both an increase in size and the formation of a purulent spot. In search of second medical opinion, he visited our out-patient clinic. Prehospital magnetic resonance imaging (MRI) indicated soft tissue swelling on the ulnar side of the left upper arm, with an internal mass-like elongated T2 signal and cellulitis-like enhancement on the enhancement imaging. He recalled no history of distant travel, animal bites or scratches. As a construction worker, he was generally well and the only significant medical history was lumbar disc herniation microdiscectomy he received 10 years ago.

On admission, the patient complained of coughing with white sputum, severe anorexia and nausea. Worse even, the mass had ruptured on the way to hospital, and he had to covered it with some gauze. During the dressing change, it was observed that the mass was swollen with a sinus tract, and approximately 15 mL exudate was drained. The exudate was initially purulent and became hemopurulent on pressure. Physical examination revealed lymphadenopathy in the unilateral axillary and supratrochlear lymph nodes, with local redness and tenderness around the abscess. Subcutaneous edema on the ulnar side of the left upper arm and forearm was observed. Lung auscultation showed scattered rales in both lungs, occasionally with wheezing. Pre-operative blood tests showed elevated white blood cell count (WBC) of 13.08*10^9^/L (normal range 4.0–10.0*10^9^/L), elevated C reactive protein (CRP) of 37.54 mg/L (normal range 0.00–8.00 mg/L) and negative result of HIV infection. Meanwhile, the patient showed no signs of fever (Temperature = 36.6 °C). Pulmonary CT scan showed inflammation on both lungs with interlobular and pleural effusion. Therefore, the patient was started empirically on intravenous infusion of piperacillin/tazobactam for the lesion and possible lower respiratory tract infection. On day 2 of admission, the first surgery was performed, where an extended incision was made to expose the subcutaneous fascia, revealing large amount of inflamed granulation tissue. The ulnar nerve was intact but adherent to surround tissue, and careful dissection was performed to free the ulnar nerve and avoid nerve damage. After excision of necrotic tissue, the abscess cavity was repeatedly irrigated and covered with vacuum sealing drainage (VSD) device. The excised tissue was then set for NGS, pathological tests and bacterial culture (Fig. 1).

**Fig. 1:** (**A)**: MRI image of the mass on admission; (**B**): Preoperative view of the mass, the pus head has ruptured; (**C)**: Intra-operative view of the mass, most necrotic or infected tissue have been removed; (**D)**: Post-operative histopathological results showing acute and chronic inflammation of subcutaneous soft tissue with histiocytes infiltration (marked by green triangle and magnification on the upper right corner), regional inflammatory granulation tissue hyperplasia (marked by red star)

In the meantime, on day 4 of hospitalization, the patient complained of shortness of breath with decreased blood oxygen saturation levels, and an urgent pulmonary CT scan was ordered. The repeated CT report showed progressed bilateral pleural and interlobar effusions with atelectasis of both lower lobes, and a new ground-glass opacity in the apical segment of the right upper lobe, suggestive of inflammatory changes. At consultation in respiratory medicine experts, bilateral thoracentesis and placement of chest drainage tubes was ordered, and a total of 1100 mL yellow clear pleural effusion was drained on the first day. The pleural drainage was collected and underwent routine, biological examination and bacterium culture, indicating Non-septic Exudative Pleural Effusion. Multiple tissue sample were sent for testing and culture, and the NGS result on day 5 reported presence of *B. henselae* in the abscess, which confirmed the diagnosis of CSD. Further inquiry on medical history revealed that the patient owned a rural warehouse where he kept clothing and bed sheets, and a pet cat, although he remembered frequent visit of local feral cats. The warehouse was relatively poor in terms of air flow, where he would take occasional naps. After alteration of antibiotic plan to doxycycline combined with azithromycin, the pulmonary distress gradually resolved and inflammatory indicators reduced to normal level on day 8 (CRP: 0.49 mg/L; WBC 5.02*10^9^/L).

On day 8 of admission, the patient reported relief from chest tightness and shortness of breath, and a repeated CT showed interstitial changes in both lungs without pleural effusion on day 8 of admission (Fig. 2). The bilateral chest drainage tubes were then removed.

**Fig. 2:** Pulmonary CT scan results with effusion indicated by red arrows. **A**: Taken 2 days prior to admission, showing interstitial changes, pneumonia with minor amount of pleural effusion; (**B)**: Taken on day 4 of admission, showing progressed pneumonia with increased pleural effusion; (**C)**: Taken on day 8 of admission, showing alleviated pneumonia, and previous pleural effusion absorbed; (**D)**: Taken 2 weeks after discharge with normal result

Meanwhile, as the pulmonary symptoms relieved, the patient underwent secondary debridement, which showed localized inflammation and limited residual granulation tissue, and the remaining necrotized tissue was removed before suturing. The patient was generally well after the second surgery and discharged on day 11 of admission.

On out-patient follow-up 2 weeks later, the patient recovered from the previous symptoms. Physical examination showed negative pulmonary signs, and the incision healed without further inflammation.

## Discussion

CSD has been reported to cause pleural effusion possibly due to obstructed lymphatic drainage from the lungs [19]. In this case, the pulmonary CT scan on day 4 of admission showed interstitial inflammation with bilateral pulmonary effusion, indicating a possible role of COVID infection. This phenomenon was also observed in canine, as reported by Cherry N. et al. in 2009 [20]. Interestingly, a canine study led by Weeden A. et al. indicated positive *B. henselae* DNA in pleural and peritoneal effusion while pericardial effusion showed negative results [21]. In our case, the recurrence of localized mass and subsequent pleural effusion was parallel to COVID infection, possibly due to disrupted immune response.

As a zoonotic pathogen, *B. henselae* is transmitted to cats by flea feces contamination and ingested while grooming, therefore transmission to human is often achieved by cat scratches and bites [22, 23]. This was corroborated by Chomel B. et al. in 1996, where they observed transmission of *B. henselae* to specific-pathogen-free (SPF) cats through contact with infected flea. They also noted that highly bacteremic cats, in absence of fleas, were unable to infect SPF cats [24]. The seasonality of CSD diagnosis, interestingly, has also been extensively studied by Nelson A., Saha S. and Mead P. in the United States spanning from 2005 to 2013 [25]. It was observed that the largest proportion of CSD diagnosis was made during January, followed by August and November, which they attributed to adoption pattern and age susceptibility of kittens, and peaking of fleas during fall and winter [26]. This is in line with our patient, who was also admitted in January.

In terms of source of infection, our patient denied cat scratch or bite on admission, whereas indirect contact with cats was found possible in his warehouse. The indirect mode of *B. henselae* transmission in this case was recently reported by Bush J. et al. in 2023, and they revealed the ability of *B. henselae* to exist stably in several biological and non-biological fluids [27]. While the discovery is exhilarating, the possibility of indirect *B. henselae* transmission poses a challenge for clinicians in face of similar patients without relevant history of feline contact.

Infection of *B. henselae* could cause diverse clinical symptoms depending on the age group, where children and younger individuals are prone to develop lymphadenitis while the elderly are more likely to suffer from endocarditis, and combined with *B. quintana* account for over 90% *Bartonella* endocarditis cases [28]. While it is necessary to consider infection of *Bartonella* species in the differential diagnosis in patients with fever of unknown causes, CSD is often misdiagnosed since the diagnosis is critically dependent on serological tests or polymerase chain reaction (PCR) assay as routine blood culture methods fails to detect *B. henselae* [5]. While serological test often shows high sensitivity, it fails to distinguish from ongoing infection and past infection. On the other hand, PCR assay has been shown to detect *B. henselae* in fresh tissue or purulent sample with high sensitivity and specificity, as reported by Gaoz S. et al. in 2022 [29]. The major challenge for clinicians and microbiologists is that PCR requires specific target, which is sometimes unidentified initially. Another factor for PCR sensitivity is the type of sample, since Khalfe N. and Lin D. observed decreased PCR sensitivity in paraffin embedded sample fixed by formalin [30]. In comparison, NGS could detect the species of pathogen with a quantity profile, offering assistance for clinicians to narrow down suspected pathogens at an early stage of diseases.

COVID has been characterized as a highly transmissible emerging pathogen, causing mild to severe respiratory symptoms with or without systematic complications and spreading fast across the world [31]. In context of the global pandemic of COVID, the incidence of various disease has surged due to a variety of reasons. A national study in Argentina in 2022 reported that COVID pandemic is associated with increased incidence of CSD, which was attributed to the prolonged cat contact due to quarantine, and higher rates of systematic CSD, which is yet to be explained [32].

## Conclusion

In conclusion, we present a case underscoring the importance of vigilance in diagnosing and managing unusual presentations of less common diseases, especially in the context of the COVID-19 pandemic. While CSD is typically a self-limiting condition, this case was complicated by COVID-19, leading to unique challenges in both diagnosis and treatment. The co-occurrence of these two conditions highlights the complexity of managing infectious diseases in a time of a global pandemic. Clinicians, hence, should consider multiple diagnostic possibilities and adapt treatment strategies accordingly.

## Data Availability

The dataset supporting the conclusions of this article is included with the article.
